This article has been retracted.

# Relationship of Table Tennis Sports Nutritional Food to Sports Athletes' Training and Physical Health

**DOI:** 10.1155/2021/1873312

**Published:** 2021-09-07

**Authors:** Rong Qi

**Affiliations:** Institute of Physical Education, Shanghai Normal University, Shanghai 200234, China

## Abstract

Table tennis has a broad mass base in our country and is a sport suitable for all ages. It has achieved outstanding results in the international arena and has become our country's traditional advantage. To engage in professional table tennis, table tennis players are required to have good physical quality. However, table tennis is actually a high-intensity, high-skills sport. It has a very large impact on the main power-generating parts and joints of the athlete's body. Soldiers and ball players often suffer from sports injuries. Therefore, it is necessary to carry out the nutrition corresponding supplements and targeted training. Therefore, the experimental group members were supplemented with nutritious food to distinguish the control group. The operation steps and experimental principle of this method are provided in detail in this article. Based on the above test scheme, a comparative experiment has been done and a number of physiological tests on the two groups of sports have been carried out. It includes the statistical analysis of athletes' body composition changes after the experiment and the comparative analysis of body composition before and after nutrition intervention in the experimental group. Analysis of experimental data shows that nutritional food can improve the physical indicators of table tennis players and enhance the overall health evaluation coefficient.

## 1. Introduction

Table tennis has been popular since the end of the 19th century and has a history of more than 100 years of development. Since the founding of New China, Chinese table tennis has gone through 67 years of development. At the beginning of table tennis, Japan, Europe, and other countries have always been table tennis powers, until the 1960s, Chinese table tennis formed a pen-hold close to the table with a technical style of “fast, accurate, ruthless, and change,” and it was at the forefront of the world. The advantage of table tennis transferring from Japan to China is also the second major improvement in the level of table tennis. From the 1970s to the 1980s, China's table tennis technical style had new developments. The combination of “fast, accurate, ruthless, change, and transformation” was a fast-attack combination of technical styles. The lap ball is the most prominent. In the 1990s, the technical style was mainly characterized by specialties. On the basis of the continuation of the previous technical essence after 2000, the technical requirements of Chinese table tennis are outstanding with specialties, comprehensive technology, and no obvious technical loopholes for the development direction. The innovation of technical style has brought the level of table tennis to be improved again and again, making table tennis develop into an advanced, complete, and comprehensive competitive sport.

According to GB/t24154-2009 “general principles of sports nutrition food,” sports nutrition food is a kind of food which can supplement or meet the special needs of human body for sports. This definition, proposed by the Ministry of light industry of the People's Republic of China, has a more specific explanation: in order to meet the physiological and metabolic needs of athletes and people participating in physical exercise or physical labor, and the needs of specific nutrients, food and nutritional supplements are prepared according to special formula and special treatment or preparation. According to the different needs of energy and nutrients, sports nutrition food can be divided into the following categories. (1) Energy supplement, that is, carbohydrate as the main component, can provide fast, sustained energy sports nutrition food. (2) Energy control, that is, sports nutrition food with low energy and low fat, which can meet the needs of body weight control. (3) The supplement of protein and its hydrolysate, namely, supplement protein, skin, amino acid, and its derivatives, suitable for human tissue repair, increases the demand for muscle people to eat sports nutrition food. (4) Vitamin and mineral supplement, supplement the vitamin, mineral, and sports nutrition food lost in human body exercise. (5) Supplement nutrients to eliminate exercise fatigue, that is, supplementing the nutrients to relieve the fatigue of central nervous system or peripheral body. (6) Complex nutrition, that is, sports nutrition video which can meet the basic nutritional needs of human body movement, such as sports nutrition food with replacement meal or additional meal. (7) Other categories, namely, sports nutrition food not included above. In order to improve athletes' physical fitness, the mainstream method is to supplement nutritional food. However, there is little research on table tennis players and nutrition food in China. Therefore, this paper studies the relationship between table tennis nutrition food and athletes' training and physical health. Now, people's understanding of physical health is becoming more and more thorough. Physical strength and health are related to people's physical shape, physical function, physical fitness, and psychological status. Health is a manifestation and reflection of physical fitness. Similarly, if you want to be healthy, you must first have a good physical fitness.

Physique and health are two interrelated concepts that look at the condition of the human body from different levels and categories. Regarding the research of physical fitness test items, both domestic and foreign, they attach great importance to it. First of all, this paper studies the core concepts of table tennis and nutritious food. Through the research, this paper believes that table tennis, as a high-intensity competitive sport, has high requirements for athletes' physical quality. At present, the professional table tennis training in our country often ignores the balance of diet, resulting in incomplete nutrition. However, the emergence of sports nutrition food makes up for this very good point; the reasonable use of sports nutrition food can quickly improve the physical function of exercise. Then, in order to verify the theory, this paper establishes a table tennis player's physical fitness test program about nutrition intervention. The research samples of the program are all human volunteers. In order to experience the differences of the program, the volunteers were randomly divided into two groups through multiple horizontal and vertical comparisons. The analysis of experimental data shows that intervention training with nutritional food for table tennis players can quickly improve their sports ability and keep their body healthy [1–3].

## 2. Core Concepts of Table Tennis and Nutrition

### 2.1. Table Tennis

Since the first World Championship in 1926, the rules of table tennis have been in the process of continuous improvement, which puts forward higher demands on athletes. The victory of the table tennis match is not only related to personal technical pursuit and training intensity but also related to external hardware equipment. After the 1990s, the rules of table tennis competition have undergone great changes. The International Table Tennis Federation has carried out many significant reforms, making the table tennis project develop in a more scientific and perfect direction and an indispensable and important position in the sports world [4, 5].

### 2.2. Physical Quality Characteristics of Table Tennis Players

In today's table tennis events, the most prominent features are the many changes in the landing point, the strong speed rotation, the fast conversion between offense and defense, and the wide range of control. The movement of the athletes and the quality of the technical actions are the direct causes that affect the effect of the shot. It is necessary for the athletes to make accurate judgments and effective counterattacks at the fastest speed in a very short time in order to seize the fighter and win the game. Speed, rotation, drop point, arc, and strength are the five elements of table tennis. The essence of movement is speed and rotation. The drop point and arc are external manifestations, and the root cause of table tennis is strength. The direction of the ball in the air is determined by the racket type and the direction of force; the speed of the arc and the rotation are determined by the racket type, the force of the ball, and the direction of force; and the final hitting force determines the flight speed of the ball. It can be seen that when the racket shape is in a fixed state, the final swing speed of the racket determines the final hitting power. On top of this, what determines the quality of the shot is the rapid contraction of the forearm at the moment of the shot. It can be seen that, for table tennis, the ability to efficiently complete technical movements is not only the strength generated by the upper limbs but also the coordination, cooperation, and transmission from all parts of the body [6, 7].

### 2.3. Requirements of Table Tennis Players' Physical Quality

Table tennis is an endurance load with a lower average intensity. As the duration of the load increases, so does the proportion of athletes relying on fat metabolism for energy. A large number of studies have shown that table tennis is a moderate-intensity aerobic metabolism-based sport. Table tennis is also a highly antagonistic sport, requiring athletes to have good physical qualities, such as speed, explosiveness, and coordination. Especially in recent years, the development of table tennis in the direction of high speed, high intensity, and high confrontation has put forward higher requirements on the physical fitness of table tennis players [8–10].

#### 2.3.1. Requirements of Strength and Quality

Strength quality is the guarantee of table tennis players' physical quality and the material basis for the rapid change of table tennis techniques and tactics. Modern table tennis players must be fully developed. Comprehensive strength is the strength that the players show in the coordination of various sports links in table tennis special activities. It is the basis of the special ability of the players. Improving the comprehensive strength in training is the development trend of modern table tennis strength training.

#### 2.3.2. Speed Quality Requirements

Sensitivity (the ability of the human body to quickly reposition, change movement, and adapt to changes) is very important for fast-moving ping pong balls that rotate between offense and defense. Studies have shown that sensitivity is mainly affected by the neural control of the cerebral cortex, the functional state of sensory organs, the acquisition of motor skills, and other physical health levels. Therefore, whether the strength training in the “core area” has a positive impact on the sensitivity of table tennis players is also one of the contents of this research. The distance range of the first 2 m and the rear 4 m of the “8” step test is basically the range area that the table tennis event needs to control. The athlete's ability to quickly brake, move, and accelerate within this range has a direct impact. It can be seen that, after moderate “core zone” strength training, the athlete's “core zone” strength group strength ability increases, and at the same time the athlete's “8” step speed also tends to increase.

### 2.4. Definition of Sports Nutrition Food

Sports nutrition food refers to some special food processed according to scientific methods in order to meet the nutritional needs of human body after exercise and maintain normal metabolism. In general, different types of sports foods contain much more of each nutrient than the daily dietary intake. Different types of products can meet the needs of different sports and intensity sports fitness crowd. According to the different functions and functions of nutrients contained in various nutritional foods, they can be divided into several categories. Although China's sports nutrition food market has not appeared for a long time, it has developed rapidly. The relevant market management institutions have been gradually established, and the relevant “sports nutrition food industry standard” has been issued. Various nutrients widely exist in different kinds of food, and their contents are not the same. Sports nutrition food is a special process to purify and concentrate the nutrients in food, so as to meet the needs of human body for various nutrients after exercise. Therefore, according to the different needs of physical exercise population, the use of different types and functions of sports nutrition food is conducive to people's exercise and recovery after physical exercise. Through reading the relevant literature, the author has carried on the investigation and the research in the different consumer groups and also has his own opinion to define the sports nutrition food. Sports nutrition food refers to special nutrition and health food, which contains a variety of nutrients with high purity and concentration to meet the needs of people after sports and fitness exercise [11–13].

### 2.5. Classification and Characteristics of Sports Nutrition Food

Sports nutrition products generally do not need to obtain FDA batch number, but gain market competitive advantage mainly through product formula, scientific basis, and taste and use effect. Therefore, the manufacturers increase the investment in scientific research, and the classification and serialization of products are also higher [14, 15]. According to the function of sports nutrition products, sports nutrition food can be divided into the following seven categories.

#### 2.5.1. Building Muscle Strength

Protein powder and other protein preparations that promote tissue and muscle growth and repair are the most popular sports supplements, followed by creatine. Other sports supplements include boron, chromium, Albin, colostrum, HMB, ornithine, ketoglutarate, cyclohexyl, alum, and zinc.

#### 2.5.2. Losing Weight

The most commonly used diet food is thermogenic preparation, which usually contains caffeine, ephedrine, aspirin, etc. In particular, L-carnitine, which promotes the burning of fat and sugar, is widely used in people who lose weight.

## 3. Physical Fitness Test Method of Nutrition Intervention

### 3.1. Research Object

The research object is a table tennis club member, including 68 men and 24 women, a total of 92 people, with the average age of 24.3 ± 1.24 years old. So, people were randomly divided into two groups, 46 people in each group. The experimental group was given nutritional intervention, and the control group was given placebo.

### 3.2. Documentation Method

We have consulted a large number of literatures and monographs closely related to this research and participated in training, nutrition, food science, physiology, sports biochemistry, pharmacology, and other disciplines. The average body weight of carbohydrate, protein, and fat and the upper and lower limits of body weight intake range were calculated according to the food nutrition table in food nutrition. The energy produced by the three nutrients is converted according to the food equivalent exchange table and food energy coefficient in sports nutrition. According to the recommended intake of three nutrients for sprinters in “Recommended Dietary Nutrients and Appropriate Dietary Intake for Chinese Athletes,” this paper analyzes the ratio of energy output to output of three nutrients for table tennis players. According to the survey results, the productivity ratio of each meal was calculated and compared with the recommended energy supply ratio of three meals a day.

### 3.3. Questionnaire Survey

KAP questionnaire is based on the needs of the study to understand the nutritional knowledge, attitude, and behavior of the participants. The dietary behavior of athletes is closely related to their knowledge and attitude. According to the theory of knowledge, attitude, and behavior, knowledge (information) is a necessary condition for behavior change. Belief (attitude) reflects behavior tendency. To change behavior, attitude is the first thing to change. KAP survey results of athletes have important reference value for the research of athletes' basic diet problems and the application of nutritional supplements. The questionnaire design of KAP is based on the relevant information needed to obtain in this subject. On the basis of a large number of references, drawing on the content and mode of KAP questionnaire developed by predecessors, a questionnaire on table tennis players' nutrition knowledge, attitude, and behavior was developed.

The 24-hour dietary review is an important method of data collection. In the process of investigation, athletes were included in the survey, including the names of meals and snacks, meals, food intake, and detailed records. As a subject of research, the analysis of athletes' dietary structure and the proportion of the three major nutrients provide raw data. The article experiment uses logical analysis to describe the information displayed by the data in concise and rigorous language to make people clear at a glance. At the same time, the main factors affecting the healthy development of students' physical fitness are found through logical analysis, and the experiment is true and reliable.

### 3.4. Reliability and Validity of KAP Questionnaire

A questionnaire survey was conducted on 92 athletes. 60 athletes were randomly selected and this was repeated every 15 days to test the reliability and validity of the questionnaire. The consistency of basic nutrition knowledge, attitude, and behavior was 0.89, 0.93, and 0.95, respectively, and Pearson correlation coefficient was statistically significant (*P* < 0.05).

### 3.5. Nutrition Supplement Program

This paper discusses the measures of strengthening and recovering after large amount of exercise from various stages before, during, and after exercise. The main measure of nutrition recovery is to eliminate the bad factors and balance the internal environment that is to achieve the balance of water, salt, and acid-base. The nutrition loss after exercise training includes body fluid, energy reserve, and active protein. At the same time, it can stimulate the secretion of synthetic hormone, repair the anabolism, renew the tissue, and improve the function. According to the above principles, the nutritional supplement program is formulated, as shown in Table 1.

### 3.6. Aerobic Exercise Ability Test

Aerobic capacity refers to the ability of the body to provide energy for the body through aerobic oxidation, so as to maintain exercise. Aerobic capacity refers to the comprehensive ability of human body to absorb, transport, and utilize oxygen. It refers to the ability of the human body to absorb oxygen in the body per unit time, transport oxygen through blood circulation, and be absorbed into the activity of muscle tissue.

After comprehensive consideration, this study used the 15-minute running test to evaluate the aerobic ability of athletes and record the running distance. In EKF Biosen C, Germany, with the help of glucose/lactate analyzer, finger blood was collected before and after exercise, and blood lactic acid was measured.

### 3.7. Anaerobic Exercise Ability Test

The anaerobic capacity of athletes was tested by 30 s Wingate test. The basic principle of the test is that the 30-second exercise is mainly based on the energy provided by glycolysis. The more work the subjects complete in the test process, the stronger their glycolysis ability. Test steps: (1) athletes ride powered bicycles for 3–5 minutes, and their heart rate increases to 140–150 beats/min. There were 3–4 full intensity rides in the middle, each time about 5–10 seconds. (2) Rest for 5–8 minutes. (3) Formal test: after issuing the riding password, the weight of the tested athlete reaches the preset value within 3–5 seconds, and then the number of cycling laps is recorded. The athlete insists on riding fast for 30 seconds, and the recording frequency is 2 times and 10 seconds. The heart rate and speed are recorded.

## 4. Experimental Results and Analysis

### 4.1. Analysis of the Characteristics of Body Function

As can be seen from Figure 1, before the “nutritional supplement” experiment, the difference of “health assessment score” between the experimental group and the control group was only about 1 point. In addition, in most other indicators, such as weight, skeletal muscle, percentage of body fat, and heart rate index, the difference was not significant. There was no significant difference in blood glucose and blood lactate between the two groups before and after exercise. There was no significant difference between the experimental group and the control group before the nutritional intervention, indicating that the physiological indexes of the two groups of athletes were basically maintained at the same level before the intervention, which can be compared with the next step of experimental intervention.

### 4.2. Statistical Analysis of Changes in Body Composition of Athletes

Compared with Figures 1 and 2, it can be seen that the improvement degree of the health evaluation score of the experimental group is higher than that of the control group, indicating that, after four weeks of experimental intervention, the health status of the athletes has slightly improved. After comparing the body composition, it was found that the weight gain rate of the test group and skeletal muscle was higher than that of the control group, and the growth rate of body fat and the percentage of body fat in the test group were lower than those in the control group. Four weeks after the experiment, the body composition of athletes had a benign change. These data can directly reflect the positive impact of nutrition supplement on the body composition and body formation of athletes.

### 4.3. Comparative Analysis of Body Composition before and after Nutritional Intervention in the Experimental Group

From the statistical results of Figures 2 and 3, it can be seen that the weight of the players increased significantly after nutrition intervention, and at the same time, the overall health evaluation of football players was improved compared with that before the experiment. The specific performance is skeletal muscle content increased significantly, and the percentage of body fat increased, indicating that nutritional intervention has a positive impact on the body shape of table tennis players in the experimental process. Only in terms of weight, compared with before the experiment, the weight of all subjects was basically stable in the whole experiment. The growth rate is in line with the natural development law of the human body, indicating that the energy supply of nutritious food basically meets the demand growth and the competition of development and training, and the content of protein and fat does not exceed the standard.

### 4.4. Statistical Analysis on Physiological Indexes of Athletes after Intervention

Independent sample *t*-test and paired sample test were used to compare the physiological changes of the two groups after four weeks of nutrition intervention. The results of Figure 4 and Table 2 show that the body composition and changes of each group before and after the experiment are significant. After 4 weeks of nutritional intervention, the indexes of blood lactic acid and core muscle strength in the experimental group were significantly different, but there was no significant difference in the physiological indexes of the control group. The cardiac function index and muscle strength of each group were significantly improved, but the difference was not statistically significant. After 4 weeks of intervention, there was no significant difference in physiological indexes between the experimental group and the control group, indicating that the nutritional supplement has a certain promoting effect on table tennis players.

## 5. Conclusions

Table tennis is a traditional sport in our country, and most athletes fight alone or play against each other. Due to its small size, fast speed, many changes, and complicated techniques, table tennis requires higher physical fitness during the game. And for the training of table tennis players, traditional training methods have shown certain shortcomings, and scientific training programs have not been customized according to the characteristics of the players themselves. While strengthening the training intensity, it also exposes some basic problems such as the athlete's physical quality not keeping up with it. But at present, there are too many studies on this problem in China. Therefore, the research on the relationship between table tennis sports nutrition food and sports athletes' training and physical health proposed in this paper can make up for the deficiency in this field. The scheme of this paper is to adopt the current mainstream nutritional food supplement method, which has been widely used in many competitive sports fields and has achieved ideal results. In order to verify the practical effectiveness of this method in table tennis players training, this paper established the relevant nutrition intervention test model. The model can improve the performance of athletes by changing diet habits and adding minerals. At the same time, in order to test the effect, in addition to the experimental group, we also set up a control group, which is convenient for horizontal and vertical comparison. At the end of this article, a comparative experiment is carried out by statistical analysis of the physiological indicators of the table tennis players after the intervention. Compared with the experimental data analysis, after four weeks of nutritional intervention, the physical and physiological indexes of table tennis players in the experimental group were significantly improved. And through the comparison with the control group, there are obvious differences, so this paper believes that the intake of nutritional food can effectively improve the sports ability of table tennis players. All sectors of society should actively cooperate with related activities to improve the physical health of athletes. Only in this way can the athlete's physical fitness level get a qualitative leap.

## Figures and Tables

**Figure 1:** Analysis of table tennis players' physical function before and after the experiment.

**Figure 2:** Statistical analysis of the changes of athletes' body composition after the experiment.

**Figure 3:** Comparative analysis of body composition before and after nutritional intervention in the experimental group.

**Figure 4:** Statistical analysis of physiological indexes of table tennis players after intervention.

**Table 1:** Nutrition supplement plan of this experiment.

Stage	Nutrition	Consumption	Usage
Breakfast	Whey protein	1 scoop (15 g)	Add milk to drink
	Sports drinks	650 ml	Direct drinking
General training	Electrolyte effervescent tablets	2 tablets	Add water
	Sports drinks	250 ml	Direct drinking
Big training	High magnesium tolerance	2 spoons (15 g)	Add drinks
	Sports drinks	250 ml	Direct drinking
Before big training	Creatine powder	1 scoop (10 g)	Add milk to drink
	Strong joint	2 capsules	Add water
	Powerful antioxidant	2 capsules	Add water
	Whey protein	1 scoop (15 g)	Add drinks
After a lot of training	Active sugar capsule	10 capsules	Peel and add to drink
	Glutamine Q	10 capsules	Peel and add to drink
After dinner	Haematol	4 capsules	Add water
	Calcium magnesium D	3 capsules	Add water

**Table 2:** Statistics of physiological indexes of athletes after intervention.

Index	Experience group	Control group	*t*	*P*
Blood glucose before exercise (A)	5.48 ± 4.85	3.41 ± 2.16	0.95	0.33
Blood lactic acid before exercise (B)	5.69 ± 0.104	6.12 ± 0.83	−1.24	0.14
Blood glucose after exercise (C)	7.99 ± 2.82	7.21 ± 3.35	0.08	0.87
Blood lactic acid after exercise (D)	5.49 ± 1.49	4.85 ± 1.29	0.19	0.96
Heart work index (E)	16.35 ± 5.36	17.83 ± 4.47	−0.27	0.87
Heart rate index (F)	23.96 ± 2.85	24.87 ± 3.36	−0.31	0.75

## Data Availability

The data that support the findings of this study are available from the corresponding author upon reasonable request.
